# miR-18a-5p Facilitates Malignant Progression of Head and Neck Squamous Cell Carcinoma Cells via Modulating SORBS2

**DOI:** 10.1155/2021/5953881

**Published:** 2021-10-18

**Authors:** Qian Chen, Jing Xu, Mingzhen Zhu

**Affiliations:** Department of Oncology, The Second People's Hospital of Lianyungang (The Oncology Hospital of Lianyungang), Lianyungang City, Jiangsu Province 222000, China

## Abstract

This study attempted to investigate possible molecular mechanism and role of miR-18a-5p in head and neck squamous cell carcinoma (HNSCC). Differential miRNAs and their possible targets were analyzed through TCGA database. By conducting qRT-PCR, miR-18a-5p was tested to be increased and SORBS2 was assessed to be downregulated in HNSCC cells. CCK-8, Transwell, and flow cytometry assays disclosed that miR-18a-5p facilitated HNSCC cell proliferation, migration, and invasion and repressed cell apoptosis. By dual-luciferase reporter gene assay, it was verified that miR-18a-5p had binding sites into SORBS2. Rescue experiments displayed that forced expression of SORBS2 restored the impact of miR-18a-5p overexpression on HNSCC cells. Collectively, our research preliminarily identified the promotion effect of miR-18a-5p/SORBS2 axis on malignant phenotypes of HNSCC cells. Our findings may provide a preclinical reference for HNSCC treatment.

## 1. Introductions

According to the statistics of GLOBOCAN, the proportion of head and neck cancer- (HNC-) related deaths to cancer-related deaths is much higher than its incidence as of 2020 [1]. Most of the tumors in head and neck areas are head and neck squamous cell carcinoma (HNSCC) which takes up nearly 90%. HNSCC is derived from epithelial cells in the mucosa of the upper respiratory tract and esophagus (oral cavity, oropharynx, larynx, and hypopharynx) [2]. Though undergoing primary radical therapies like surgery, concurrent chemoradiotherapy, or radiotherapy alone, patients with HNSCC still suffer from local reoccurrence and tumor metastasis. For patients who cannot undergo radical therapies, chemotherapy alone is not effective enough [3]. Therefore, the exploration of novel and efficient therapies is of great importance to reduce the reoccurrence rate of HNSCC.

Anomalous changes in miRNA expression profile are ubiquitous phenomena in various tumors. Researchers analyzed miRNA expression profile in breast cancer tissue and then discovered 121 differentially expressed miRNAs (DE-miRNAs) utilizing microarray approach [4]. In addition, abnormity of miRNA expression profile also exists in all kinds of tumor tissues like lung adenocarcinoma, liver cancer, oral cavity squamous cell carcinoma, and colorectal cancer. There are increasing studies on the effects of miRNA on HNSCC. For example, miR-150-5p and miR-150-3p suppress invasion of cancer cells via binding to SPOCK1 in HNSCC. Besides, overexpressing miR-642b-3p dramatically reduces migratory and invasive properties of HNSCC cells and upregulates apoptosis ability [5]. As an important member of miRNA family, miR-18a-5p strengthens radiosensitivity of lung cancer stem cells by decreasing the expressions of ATM and HIF-1*α* in recent years [6]. Based on the increased miR-18a-5p expression in renal cell carcinoma (RCC) tissue and cell line, further studies revealed that increased miR-18a-5p positively modulates malignant phenotypes of RCC cells. However, downregulation of miR-18a-5p neutralizes such effect, which shows that miR-18a-5p serves as an oncogene and prognosis biomarker in RCC [7]. miR-18a-5p directly targets IRF2 to promote the invasion and migration of osteosarcoma [8]. It also targets SPEBP1 to form inhibitory complex with Snail and HDAC1/2to modulate epithelial-mesenchymal transition (EMT) of breast cancer [9]. Nevertheless, it is poorly studied in HNSCC.

SORBS2 can interact with actin and some cytoskeletal proteins [10]. In the existing studies, SORBS2 serves as a repressor in cancers, such as suppression on the invasion of ovarian cancer cells [11] and proliferation, invasion, and migration of liver cancer cells *in vivo* and *in vitro* [12]. To date, there is no study on the effect of SORBS2 on HNSCC.

This study displayed that the miR-18a-5p level was markedly upregulated in HNSCC by analyzing profiles from The Cancer Genome Atlas (TCGA) database. Furthermore, we predicted downstream target gene to reveal binding of miR-18a-5p and SORBS2. Next, we investigated modulatory mechanism of miR-18a-5p/SORBS2 in HNSCC, which provides new basis to elucidate the molecular mechanism of migration and invasion of HNSCC. Meanwhile, we offer novel targets for the treatment of HNSCC and further reveal the close connection between miR-18a-5p and malignant progression of HNSCC.

## 2. Materials and Methods

### 2.1. Bioinformatics Approaches

miRNA mature expression data and total RNA sequencing data of HNSCC were obtained from TCGA (https://portal.gdc.cancer.gov/) database. After screening the data, we obtained 518 cancer tissue samples and 44 normal tissue samples from miRNA data. We also obtained 495 cancer tissue samples and 44 normal tissue samples from total RNA sequencing data. Afterwards, the miR-18a-5p level was identified and DE-mRNAs were identified via R package “edgeR” (∣logFC | >2, padj < 0.05). After miRNAs were determined, likely targets of miRNA were identified via TargetScan (http://www.targetscan.org/vert_72/), mirDIP (http://ophid.utoronto.ca/mirDIP/), miRDB (http://mirdb.org/), and starBase (http://starbase.sysu.edu.cn/) databases, and were overlapped with DE-mRNAs. Finally, correlation between miRNAs and mRNAs was analyzed and miRNA-mRNA regulatory pairs were determined.

### 2.2. Cell Culture

Immortal human keratinocytes HaCaT were accessed from Cell Resource Center, Institute of Basic Medicine, Chinese Academy of Medical Sciences. FaDu (BNCC316798), SCC-9 (BNCC250260), SCC-15 (BNCC275715), and SCC-25 (BNCC315876) were all human HNSCC cell lines and were bought from BeNa Culture Collection (BNCC). They were maintained in DMEM with 10% fetal bovine serum (FBS) and hydrocortisone (400 ng/mL). HaCaT cells were incubated in MEM-EBSS with 15% FBS. FaDu cells were maintained in Eagle's MEM (No. 30-2003) (American Type Culture Collection (ATCC)) with 10% FBS. Culture condition was an incubator with 5% CO_2_ at 37°C. After infusion degree of cells reached 80%, they were used for subculture or assays.

### 2.3. Cell Transfection

miR-18a-5p-mimic (miR-mimic), negative control NC-mimic, pcDNA3.1-SORBS2 (oe-SORBS2), and pcDNA empty plasmid (oe-NC) were purchased from GenePharma (Shanghai, China). As guided by instructions of manufacturer, miR-18a-5p-mimic, NC-mimic, and plasmids were transiently transfected into SCC-15 cell line utilizing Lipofectamine 1800 (Invitrogen, Carlsbad, CA). Thereafter, cells were maintained for 2 days in mediums with 5% CO_2_–95% air at 37°C for study.

### 2.4. qRT-PCR Assay

Total RNA was isolated from HNSCC cells with TRIzol kit (Life Technologies, NY, USA) in adherence to instruction. MiScript IIRT kit (Qiagen, Dusseldorf, Germany) and PrimeScript RT Master Mix (Takara, Dalian, China) were applied to reversely transcribe miRNA and mRNA into cDNA, respectively. MiScript SYBR Green PCR kit (Qiagen, Dusseldorf, Germany) and SYBR® Premix Ex Taq™ II (Takara Bio Inc., Shiga, Japan) were separately used to detect miRNA and mRNA levels. Applied Biosystems® 7500 Real-Time PCR Systems (Thermo Fisher Scientific, Waltham, MA) was employed to perform qRT-PCR assay. GAPDH and U6, respectively, served as references for SORBS2 and miR-18a-5p. Difference in relative expression was compared by the 2^-*ΔΔ*Ct^ value. Primer sequences are listed in Table 1.

### 2.5. Western Blot Assay

Western blot is an assay that tests the relative expression of proteins via 3 approaches: SDS-PAGE, western blotting, and enzyme immunoassay. Here are the detailed processes. Firstly, cells were lysed to prepare protein samples. Protein extracts were isolated with 10% SDS-PAGE, and then, proteins were transferred to a PVDF membrane. Afterwards, membrane was incubated at 4°C with primary antibodies overnight: rabbit anti-SORBS2 (1 : 100, ABIN5553826, Antibodies, US) and rabbit anti-GAPDH (1 : 10000, ab181602, Abcam, Cambridge, UK) and followed by 2 h incubation with secondary antibody goat anti-rabbit IgG H&L (ab6721, Abcam, Cambridge, UK). Finally, with GAPDH as the internal reference, ECL kit (GE Healthcare, Chicago, USA) was used to test the expression of proteins.

### 2.6. CCK-8 Assay

Posttransfected HNSCC cells were plated into a 96-well plate (4 × 10^3^ cells/well). Each well was added with CCK-8 solution (10 *μ*L/well) in days 1, 2, 3, and 4. Samples were maintained at 37°C for 2 h. Optical density at 450 nm was assayed with a microplate reader (Bio-Rad Laboratories, CA, USA).

### 2.7. Cell Migration and Invasion Assays

A Transwell chamber (BD Biosciences, CA, USA) was inoculated with transfected cells (5 × 10^4^ cells/well), and a lower chamber was supplemented with cell mediums plus 10% FBS. At 48 h after being cultured at 37°C, cells that remained on the top of the membrane were discarded. Other cells were fixed with 70% ethyl alcohol and dyed with 0.1% crystal violet. A light microscope was implemented to observe dyed cells, and those in 5 random areas were counted for statistical analysis (magnification: 100x). Cell invasion assay was conducted in a similar way, apart from the first step in cell invasion assay that the upper room was added with Matrigel (BD Biosciences, CA, USA).

### 2.8. Cell Apoptosis Assay

To analyze cell apoptosis, transfected cells cultured for 48 were collected. In line with the instructions of the manufacturer, FITC cell apoptosis assay kit (BD Pharmingen, CA, USA) was applied to determine cell apoptosis rate. In the end, a FACSCalibur flow cytometer (Becton Dickinson, CA, USA) was implemented to assay cell apoptosis.

### 2.9. Dual-Luciferase Assay

To confirm that miR-18a-5p targets SORBS2 3′UTR, we constructed dual-luciferase reporter plasmid psiCHECK-SORBS2 (Sangon Co., Ltd., Shanghai, China) 3′-untranslated region (UTR) wild-type (wt-SORBS2) and SORBS2 3′UTR mutant (mut-SORBS2). Following the specification of Lipofectamine 2000 kit (Invitrogen, CA, USA), psiCHECK-SORBS2 wt/mut and miR-18a-5p-mimic/NC-mimic were cotransfected to SCC-15 cell. Dual-Luciferase Reporter Assay System (Promega, WI, USA) was implemented to measure viability of luciferase. Assays above were repeated in triplicate.

### 2.10. Statistical Analysis

GraphPad Prism 6.0 (La Jolla, CA, USA) was employed to analyze all of the data from three independent assays. Results were expressed as the mean ± SD, and a *t*-test was conducted between two groups. *p* < 0.05 indicated remarkable statistical significance.

## 3. Results Analysis

### 3.1. miR-18a-5p Is Increased in HNSCC Cells

We performed bioinformatics analysis via TCGA database to filter out quantities of DE-miRNAs in normal tissue and HNSCC tissue. The miR-18a-5p level was markedly high in HNSCC tissue (Figure 1(a)). Differences in miR-18a-5p level between normal cell line and human HNSCC cell lines were tested using qRT-PCR method. This assay further verified that the miR-18a-5p level in HNSCC cell lines was markedly high, compared when it was in normal cell line (Figure 1(b)).

The outcomes above demonstrated that the miR-18a-5p level was dramatically increased in HNSCC cell lines. Among various HNSCC cell lines, miR-18a-5p expression in SCC-15 cell line was the highest. We therefore chose SCC-15 cells for subsequent biologically functional assays.

### 3.2. Overexpressed miR-18a-5p Acts as an Oncogenic Gene in HNSCC

Based on remarkably increased miR-18a-5p in HNSCC cells and bioinformatics analysis on HNSCC performed in TCGA database, we manifested that the miR-18a-5p level was noticeably high in HNSCC tissue relative to that in normal tissue. This outcome denoted that miR-18a-5p exerted an oncogenic effect. To further understand the functions of miR-18a-5p on HNSCC, we constructed miR-18a-5p mimic plasmid to transfect cells. Afterwards, overexpression efficiency of miR-18a-5p to SCC-15 cells was assayed via qRT-PCR. The result exhibited that the miR-18a-5p level in the overexpressed group was dramatically higher than it was in control group (Figure 2(a)). miR-18a-5p mimic thereby could be utilized for the follow-up assays. Next, we performed CCK-8 assay to test influence of overexpressed miR-18a-5p on viability of HNSCC cells SCC-15. After miR-18a-5p was overexpressed, cell viability of SCC-15 cell was dramatically enhanced (Figure 2(b)). Subsequently, the result of Transwell indicated that the migratory and invasive speeds of SCC-15 cell in the miR-18a-5p mimic group were remarkably faster than that in the NC mimic group when enforced expression of miR-18a-5p confirmed that miR-18a-5p could serve as an oncogene in HNSCC cells (Figures 2(c) and 2(d)). Moreover, we applied flow cytometry to evaluate the impact of overexpressed miR-18a-5p on the apoptosis of SCC-15 cells. The result showed that the apoptotic rate of SCC-15 cells was noticeably lower in the miR-18a-5p mimic group relative to the NC mimic group. Overexpressed miR-18a-5p could suppress the apoptosis of HNSCC cells (Figure 2(e)). The results above demonstrated that forced expression of miR-18a-5p accelerated malignant progression of HNSCC.

### 3.3. miR-18a-5p Hinders SORBS2 Level in HNSCC Cells

We firstly analyzed the differential expressions of genes and obtained 2008 significantly and differentially expressed genes, among which 1130 genes were upregulated while 878 were remarkably downregulated (Figure 3(a), FDR < 0.05). We further employed miRDB, TargetScan, mirDIP, and starBase databases to identify likely targets of miR-18a-5p. And then, they were intersected with upregulated genes to obtain 2 candidate target genes (Figure 3(b)). Correlation analysis denoted that negative association between miR-18a-5p and SORBS2 was the strongest (Figure 3(c)). In addition, TCGA data result demonstrated that SORBS2 was markedly lowly expressed in cancer tissue (Figure 3(d)). There were significant differences of SORBS2 in patients with different T stages (Supplementary Figure 1). Hence, we selected SORBS2 as the object for the following study. Moreover, we utilized bioinformatics databases to assess possible binding sites of miR-18a-5p and SORBS2 3′UTR (Figure 3(e)). Besides, we performed dual-luciferase assay to ascertain binding between miR-18a-5p and SORBS2. miR-18a-5p upregulation dramatically suppressed luciferase activity of wt SORBS2 3′UTR while it had no such impact on that of mutant type (Figure 3(f)). Furthermore, we applied qRT-PCR to examine SORBS2 mRNA expression in different groups of SCC-15 cell line and the outcome showed that overexpressed miR-18a-5p would conspicuously inhibit SORBS2 mRNA level in HNSCC cells (Figure 3(g)). The result in Western blot also revealed that the notable decrease in the SORBS2 protein level after miR-18a-5p was overexpressed (Figure 3(h)). The above results proved the repressive impact of miR-18a-5p on the SORBS2 level in HNSCC cells.

### 3.4. miR-18a-5p Decreases SORBS2 to Accelerate Migration and Proliferation of HNSCC Cells and Hinders Apoptosis

We constructed overexpressing miR-18a-5p cell line (miR-mimic+oe-NC) and simultaneously overexpressed cell lines of SORBS2 and miR-18a-5p (miR-mimic+oe-SORBS2) to verify the impact of miR-18a-5p and SORBS2 on the biological functions of HNSCC cells. In qRT-PCR assay, we examined the SORBS2 level in transfected cells. The SORBS2 level was decreased in cell line when miR-18a-5p was overexpressed, while SORBS2 expression was restored when SORBS2 and miR-18a-5p were overexpressed simultaneously (Figure 4(a)). The outcomes in CCK-8 assay exhibited that enforced expression of miR-18a-5p enhanced the viability of HNSCC cells, but simultaneous forced expression of SORBS2 and miR-18a-5p reduced such enhanced effect (Figure 4(b)). Cell immigration and invasion assays demonstrated that enforced expression of miR-18a-5p enhanced migratory and invasive ability of HNSCC cells, while simultaneous forced expression of SORBS2 and miR-18a-5p would reduce such effect (Figures 4(c) and 4(d)). The result of flow cytometry revealed that overexpressing miR-18a-5p weakened apoptotic capacity of HNSCC cells, while concurrently enforcing expression of miR-18a-5p and SORBS2 would hinder such effect (Figure 4(e)). Thus, miR-18a-5p targeted SORBS2 expression to accelerate malignant behaviors of HNSCC cells.

## 4. Discussion

Studies on HNSCC showed the aberrant expression of various miRNAs. For example, the two strands of miR-99a-duplex (miR-99a-5p: the guide strands, and miR-99a-3p: the passenger strands) [13] and miR-876-5p [14] were lowly-expressed in HNSCC, while miR-125a-5p [15] and miR-1275 [16] were highly expressed. All of the above miRNAs are implicated in HNSCC progression. Because miR-18a-5p has a similar effect on other cancers and it is poorly studied in HNSCC, it is selected for study. Besides, miR-18a-5p high expression in HNSCC tissue was revealed by a bioinformatics method, and this result was the same with that in the subsequent qRT-PCR assay. Our study unprecedently pointed out that the miR-18a-5p level is activated in HNSCC tissue and cells.

miR-18a-5p fosters progression of all kinds of cancers. For instance, its upregulation has a positive effect on malignant phenotypes of HNSCC cells [7]. miR-18a-5p also facilitates cell proliferation and migration in lung cancer and hinders their apoptosis [17]. In recent years, miR-18a-5p was proved to enhance radiosensitivity of stem cells by downregulating ATM and HIF-1*α* in lung cancer [6]. Besides, it directly targets IRF2 to promote the invasion and migration of osteosarcoma cells [8]. Moreover, it modulates EMT of breast cancer by targeting SPEBP1, Snail, and HDAC1/2 to form inhibitory complex [9]. We overexpressed miR-18a-5p in HNSCC cell line SCC-15 to confirm that this process would result in the acceleration of proliferation and migration and repression of apoptosis in HNSCC cells. Finally, we verified that miR-18a-5p also acted as a promoter to facilitate HNSCC progression.

A great deal of studies proved that miR-18a-5p has multiple downstream genes. Zheng et al. [18] pointed out that miR-18a-5p can target CDK19 in breast cancer. Besides, Zhang et al. [19] proposed that RUNX1 is targeted by miR-18a-5p in malignant melanoma. So far, there is no literature revealing the downstream target of miR-18a-5p in HNSCC. This study used R package “edgeR” to determine differentially expressed genes in TCGA database and utilized mirDIP, TargetScan, starBase, and miRDB databases to assess likely target genes of miR-18a-5p. They were then overlapped with differentially expressed genes for the analysis of correlation between miR-18a-5p and mRNAs. miR-18a-5p and SORBS2 were remarkably and negatively correlated in HNSCC. Additionally, the result of bioinformatics analysis displayed the low SORBS2 level in HNSCC. Afterwards, binding of miR-18a-5p and SORBS2 was assessed via dual-luciferase assay. In the end, we conducted qRT-PCR and western blot to prove inhibitory effect of miR-18a-5p on SORBS2 expression.

To deeply probe into the mechanism of miR-18a-5p/SORBS2 axis on HNSCC, we generated forced expression miR-18a-5p cell line and concurrently enforced expression of miR-18a-5p and SORBS2 cell line. A series biological assays confirmed that overexpressed miR-18a-5p facilitated malignant progression of HNSCC while overexpressed SORBS2 would reverse such effect. This result demonstrated that SORBS2 functioned as a repressor in HNSCC and proved that miR-18a-5p facilitated proliferative and migratory properties of HNSCC cells and hinders their apoptosis.

In short, we proved that miR-18a-5p level was increased in HNSCC. Meanwhile, overexpressed miR-18a-5p fostered proliferation and migration of HNSCC cells and repressed apoptosis. In HNSCC, we unearthed SORBS2, an effective target of miR-18a-5p, which is downregulated by miR-18a-5p to enhance proliferative and migratory ability and weaken the apoptosis capacity of HNSCC cells. The existing studies have revealed the inhibitory effect of SORBS2 in cancers. Our study illustrated the action mechanism of the miR-18a-5p/SORBS2 regulatory pathway in HNSCC to better understand the progression of HNSCC, thus offering basis for the development of novel treatments. However, the concrete mechanism is still unelucidated. Therefore, we need to further study how the signaling pathway regulates cell phenotypes, so as to discover a prognosis marker for the early-stage clinical diagnosis of HNSCC. We aim to provide foundation for the early diagnosis of HNSCC and offer alternative avenues for the treatment of this disease.

## Figures and Tables

**Figure 1:** High level of miR-18a-5p in HNSCC. (a) Box plot of differential expression of miR-18a-5p in normal and tumor groups in TCGA database, with red indicating the normal group and green indicating the tumor group. (b) qRT-PCR approach was applied to assay the difference in miR-18a-5p expression in normal immortal human keratinocytes HaCaT and human HNSCC cell lines (FaDu, SCC-9, SCC-15, and SCC-25). ∗ indicates *p* < 0.05.

**Figure 2:** miR-18a-5p facilitates the proliferation and migration of HNSCC cells and inhibits their apoptosis. (a) Overexpressed efficiency of miR-18a-5p was detected in HNSCC cell SCC-15 via qRT-PCR. (b) CCK-8 assay was carried out to test the differences in proliferative property of HNSCC cell SCC-15 between the miR-mimic group and NC mimic group after enforced expression of miR-18a-5p. (c) Transwell migration assay was employed to measure the difference in migratory rate of HNSCC cell SCC-15 between the miR-mimic group and NC mimic group after miR-18a-5p was overexpressed (100x). (d) The difference in invasive capacity of HNSCC cell SCC-15 between the miR-mimic group and NC-mimic group after the expression of miR-18a-5p assessed via Transwell invasion assay (100x). (e) Flow cytometry was utilized to examine difference in apoptosis rate of HNSCC cell SCC-15 between the miR-mimic group and NC-mimic group after miR-18a-5p was overexpressed. ∗ means *p* < 0.05.

**Figure 3:** miR-18a-5p inhibits SORBS2 level in HNSCC cells. (a) Volcano plot of DE-mRNAs in normal and tumor groups of HNSCC in TCGA database. Red: logFC > 2 and padj < 0.05, upregulated mRNAs; green: logFC < 2 and padj < 0.05, downregulated mRNAs. (b) Venn diagram of likely target genes from miR-18a-5p and DE-mRNAs. vn-genes represent mRNAs that are differentially downregulated in HNSCC. (c) Correlation analysis of miR-18a-5p and target gene mRNAs. (d) Box plot of SORBS2 level in normal and tumor groups. (e) Schematic diagram of sequence binding of SORBS2-WT, SORBS2-MUT, and miR-18a-5p. (f) Dual-luciferase assay was launched to examine luciferase viability in different groups of HNSCC cell SCC-15. (g) SORBS2 mRNA expression in HNSCC cell SCC-15 was detected in qRT-PCR assay. (h) SORBS2 protein expression in HNSCC cells was evaluated in Western blot assay. ∗ represents *p* < 0.05.

**Figure 4:** miR-18a-5p enhances the proliferation and migration of HNSCC cells and inhibits their apoptosis via downregulating SORBS2. (a) Differences of SORBS2 expression in HNSCC cell SCC-15 (NC-mimic+oe-NC, miR-mimic+oe-NC, and miR-mimic+oe-SORBS2) were assayed via qRT-PCR approach. (b) Differences in proliferative potential of cells were examined in CCK-8 assay. (c) Migratory property of cells was evaluated in Transwell migration assay (100x). (d) Invasive property of cells was tested in Transwell invasion assay (100x). (e) Flow cytometer was utilized to examine cell apoptotic rate. ∗ indicates *p* < 0.05.

**Table 1:** qRT-PCR primer sequences.

Gene	Sequences
miR-18a-5p	F: 5′-ACACTCCAGCTGGGTAAGGTGCATCTAGTGC-3′
	R: 5′-CTCAACTGGTGTCGTGGAGTCGGCAATTCAGTTGAGCTATCTGC-3′

U6	F: 5′-CTCGCTTCGGCAGCACA-3′
	R: 5′-AACGCTTCACGAATTTGCGT-3′

SORBS2	F: 5′-AATGATCGGAATCCAGAGACACT-3′
	R: 5′-AATGATCGGAATCCAGAGACACT-3′

GAPDH	F: 5′-CCTTCCGTGTTCCTACCCC-3′
	R: 5′-GCCCAAGATGCCCTTCAGT-3′

## Data Availability

The data used to support the findings of this study are included within the article. The data and materials in the current study are available from the corresponding author on reasonable request.

## Supplementary Materials

Supplementary Materials Supplementary Figure 1: expression differences of SORBS2 in HNSCC patients with different T stages. SORBS2 was differentially expressed in patients with various T stage tumors, while it was markedly decreased in patients with T3+T4 tumors compared to those with T1+T2 tumors.

## References

[1] Sung H., Ferlay J., Siegel R. L. (2021). Global cancer statistics 2020: GLOBOCAN estimates of incidence and mortality worldwide for 36 cancers in 185 countries. *CA: a Cancer Journal for Clinicians*.

[2] Leemans C. R., Snijders P. J. F., Brakenhoff R. H. (2018). The molecular landscape of head and neck cancer. *Nature Reviews. Cancer*.

[3] Łasińska I., Kolenda T., Teresiak A., Lamperska K. M., Galus Ł., Mackiewicz J. (2019). Immunotherapy in patients with recurrent and metastatic squamous cell carcinoma of the head and neck. *Anti-Cancer Agents in Medicinal Chemistry*.

[4] Peña-Chilet M., Martínez M. T., Pérez-Fidalgo J. A. (2014). MicroRNA profile in very young women with breast cancer. *BMC Cancer*.

[5] Jiang J., Zheng M., Zhang M. (2019). PRRX1 regulates cellular phenotype plasticity and dormancy of head and neck squamous cell carcinoma through miR-642b-3p. *Neoplasia*.

[6] Chen X., Wu L., Li D. (2018). Radiosensitizing effects of miR-18a-5p on lung cancer stem-like cells via downregulating both ATM and HIF-1*α*. *Cancer Medicine*.

[7] Zhou L., Li Z., Pan X. (2018). Identification of miR-18a-5p as an oncogene and prognostic biomarker in RCC. *American Journal of Translational Research*.

[8] Lu C., Peng K., Guo H. (2018). miR-18a-5p promotes cell invasion and migration of osteosarcoma by directly targeting IRF2. *Oncology Letters*.

[9] Zhang N., Zhang H., Liu Y. (2019). SREBP1, targeted by miR-18a-5p, modulates epithelial-mesenchymal transition in breast cancer via forming a co-repressor complex with Snail and HDAC1/2. *Cell Death and Differentiation*.

[10] Fredriksson-Lidman K., Van Itallie C. M., Tietgens A. J., Anderson J. M. (2017). Sorbin and SH3 domain-containing protein 2 (SORBS2) is a component of the acto-myosin ring at the apical junctional complex in epithelial cells. *PLoS One*.

[11] Zhao L., Wang W., Huang S. (2018). The RNA binding protein SORBS2 suppresses metastatic colonization of ovarian cancer by stabilizing tumor-suppressive immunomodulatory transcripts. *Genome Biology*.

[12] Han L., Huang C., Zhang S. (2019). The RNA-binding protein SORBS2 suppresses hepatocellular carcinoma tumourigenesis and metastasis by stabilizing RORA mRNA. *Liver International*.

[13] Okada R., Koshizuka K., Yamada Y. (2019). Regulation of oncogenic targets by miR-99a-3p (passenger strand of miR-99a-duplex) in head and neck squamous cell carcinoma. *Cells*.

[14] Dong Y., Zheng Y., Wang C. (2018). MiR-876-5p modulates head and neck squamous cell carcinoma metastasis and invasion by targeting vimentin. *Cancer Cell International*.

[15] Jin S., Liu M.‑. D., Wu H. (2018). Overexpression of hsa-miR-125a-5p enhances proliferation, migration and invasion of head and neck squamous cell carcinoma cell lines by upregulating C-C chemokine receptor typeï¿½7. *Oncology Letters*.

[16] Liu M. D., Wu H., Wang S. (2018). MiR-1275 promotes cell migration, invasion and proliferation in squamous cell carcinoma of head and neck via up-regulating IGF-1R and CCR7. *Gene*.

[17] Liang C., Zhang X., Wang H. M. (2017). MicroRNA-18a-5p functions as an oncogene by directly targeting IRF2 in lung cancer. *Cell Death & Disease*.

[18] Zheng P., Dong L., Zhang B. (2019). Long noncoding RNA CASC2 promotes paclitaxel resistance in breast cancer through regulation of miR-18a-5p/CDK19. *Histochemistry and Cell Biology*.

[19] Zhang Y., Qian W., Feng F. (2019). Upregulated lncRNA CASC2 may inhibit malignant melanoma development through regulating miR-18a-5p/RUNX1. *Oncology Research*.

